# Effects of Staged Nursing Care on Neuroendoscopic Transsphenoidal Pituitary Adenoma Resection and Postoperative Complications

**DOI:** 10.1155/2022/2171529

**Published:** 2022-08-05

**Authors:** Yaya Fei, Jiajia Zhang, Yudan Gu

**Affiliations:** The Second Ward of Neurosurgery, Affiliated Hospital of Nantong University, Nantong, Jiangsu, China

## Abstract

**Objective:**

The purpose of this study was to determine whether staged nursing had an impact on the outcome of neuroendoscopic transsphenoidal pituitary tumor resection and postoperative complications.

**Methods:**

As research participants, we chose 88 individuals with pituitary adenomas who were treated at our institution between February 2020 and November 2021; all patients received endoscopic transsphenoidal pituitary adenoma excision. The patients were randomly divided into two groups: the routine group (*n* = 44) and the stage group (*n* = 44). Patients in the routine group received care according to the routine nursing mode, and patients in the stage group received care according to the stage nursing mode. The staged nursing interventions included preoperative, intraoperative, and postoperative nursing. Postoperative recovery-related indicators such as the self-rating anxiety scale (SAS) and a self-rating depression scale (SDS), contentment, comfort, and postoperative complications were compared between the two groups.

**Results:**

The postoperative recovery-related indexes of patients in the stage group were significantly lower than those in the routine group (*P* < 0.05); the SAS and SDS scores in the stage group after treatment were significantly lower than those in the routine group (*P* < 0.05); patients in the stage group were significantly more satisfied with their treatment after treatment than those in the routine group (*P* < 0.05); patients in the stage group were significantly more comfortable after treatment than those in the routine group (*P* < 0.05); a significantly lower incidence of postoperative complications was observed in the stage group compared to the routine group (*P* < 0.05).

**Conclusion:**

Patients with neuroendoscopic transsphenoidal pituitary tumor excision benefit greatly from staged nursing. The nursing approach may successfully assure the procedure's smooth completion, boost patients' postoperative recovery, and reduce patients' worry, despair, and other unpleasant feelings. The nursing approach may successfully increase clinical satisfaction and comfort of patients by minimizing the likelihood of postoperative problems, and it is well-suited for practical use.

## 1. Introduction

A pituitary adenoma is one of the most common intracranial benign tumors. Statistics show that its incidence is second only to glioblastoma and meningioma among intracranial tumors [1]. Among them, the prolactin-type pituitary adenoma with the highest incidence accounts for about 80% to 85%. Although pituitary adenoma is a benign tumor, clinical symptoms often seriously affect the quality of life of patients. Female patients manifested lactation, amenorrhea, and infertility; male patients manifested impotence, low libido, infertility, etc., and overgrown tumors could cause mass effects [2, 3]. A pituitary tumor is a benign tumor that is regularly discovered in the brain. This problem tends to occur in the anterior section of the pituitary gland in the sella area, and clinical investigations have shown that this disease predominantly affects young and middle-aged people. A pituitary tumor is associated with abnormal quantities of sex hormone, surrounding tissue compression, recurrent headaches, vision loss, and other compression symptoms that have adverse impacts on a patient's quality of life.

Presently, pituitary tumors are mainly treated surgically. Due to the rapid development of minimally invasive techniques and surgical instruments in China [4], the application of neuro endoscopy in transsphenoidal surgery has also increased. When compared with traditional craniotomies, neuroendoscopic transsphenoidal surgery causes less trauma to the patient's body, so postoperative recovery is more rapid, making it a more suitable procedure for elderly or frail patients [5].

In addition, there are promising treatment methods in traditional Chinese medicine (TCM), such as traditional Chinese medicine prescriptions. TCM etiology and pathogenesis of pituitary tumors are ascribed to the deficiency of kidney essence, dystrophy of the brain and marrow, mutual formation of phlegm and blood stasis, and accumulation of evil toxins. At present, the commonly used Chuening recipe treats the disease from the kidney, phlegm, and blood stasis. It can not only reduce serum prolactin and restore it to a nearly normal level but also reduce or even remove the tumor of pituitary adenoma with fewer side effects [6, 7]. Furthermore, studies have indicated that good postoperative treatment for pituitary tumors contributes immensely to disease recovery and improves the 'patient's prognosis.

During the last two decades, with the improvement of 'people's quality of life in China, nursing work has gradually evolved to become more refined, meticulous, and excellent. Staged nursing is an emerging nursing model that has many unique, creative, and holistic characteristics. This allows patients to face the follow-up treatment calmly, which is crucial to improving the prognosis of patients [8]. This study aimed to examine the effect of staged nursing on neuroendoscopic transsphenoidal pituitary tumor resection and postoperative complications.

## 2. Data and Methods

### 2.1. Participants

A total of 88 patients with pituitary tumors treated at our hospital from February 2020 to November 2021 were chosen as research subjects, and the patients were divided into two categories: routine group (*n* = 44) and stage group (*n* = 44). The randomization was carried out using an online web-based randomization tool (freely available at https://www.randomizer.org/). For concealment of allocation, the randomization procedure and assignment were managed by an independent research assistant who was not involved in the screening or evaluation of the participants. In the routine group, there were 26 males and 18 females; their ages varied from 30 to 52 years, with an average age of (41.28 ± 5.73) years; the disease duration ranged from 2 to 7 months, with an average disease duration of (4.23 ± 1.12) months. There were 28 males and 16 females in the phase group; the age ranged from 31 to 53 years, with an average age of (41.37 ± 5.82) years. The disease duration ranged from 1 to 7 months, with an average disease duration of (4.31 ± 1.20) months.

Before the commencement, the informed consent of the patients was obtained. This study protocol was approved by the hospital ethics committee (QW-LJH20200213). All procedures were in strict accordance with the guidelines of the Declaration of Helsinki.

### 2.2. Inclusion and Exclusion Criteria

#### 2.2.1. Inclusion Criteria

Patients who met the following criteria were included in this study:

- Patients who were clinically diagnosed with pituitary adenoma.
- Patients who showed various symptoms including decreased vision, fatigue, headaches, and nausea.

#### 2.2.2. Exclusion Criteria

The following patients were excluded from the study:

- Patients with other severe organ diseases were excluded from the study.
- Patients with poor compliance and poor cooperation were excluded from this study.
- Patients with infections, cardiovascular diseases, and other related diseases, with other serious medical diseases, coagulation disorders, or an abnormal mental status that prevented normal communications.

## 3. Methods

1. All patients in the routine group received routine nursing services: this included meal planning, oral care, physical sign monitoring, and health education.
2. A staged nursing model was used to intervene with patients in the stage group. Its characteristics are that nursing is divided into stages, such as preoperative, intraoperative, and postoperative, and different nursing interventions are carried out at each stage.

### 3.1. Preoperative

Nursing staff should reduce patients' blood vessel diameters before surgery for patients with nasal blood vessels [9, 10], and if the patient has symptoms such as cold and runny nose before surgery, these symptoms should be controlled, and the patient's condition stabilized before surgery. When the patient is sent to the operating room, the operating room's temperature and humidity should be adjusted in time, and the nurses should be kept as silent as possible during the operation. The nursing staff must test all the instruments used before the operation and ensure that the instruments used during the procedure are in a sterile state when they are used [11].

Nurses should also provide appropriate psychological care to patients before surgery. In spite of the fact that pituitary tumor disease has no major impact on the prognosis of patients, patients remain prone to anxiety, tension, and other negative emotions that affect their sleep quality, such as preoperative panic and fear for the safety of surgery, which will adversely affect their quality of sleep. Therefore, the nursing staff should provide a certain level of psychological counseling to the patient before the operation, explain to the patient the reliability of the operation and the dangers associated with pituitary tumor disease, and allow the patient to maintain a positive preoperative attitude. This will facilitate the patient's cooperation during the operation [12].

### 3.2. Interoperative

During the course of the operation, in addition to the cooperation of the equipment nurses, the circuit nurses must also be cooperative. During preoperative inspections, roving nurses should be present. As soon as the patient enters the operating room, the nursing staff should assist the anesthesiologist in performing general anesthesia and tracheal intubation and monitoring the patient's vital signs. After anesthesia, the nursing staff should pay attention to protecting the patient's eye mask and may apply appropriate eye ointment to the patient's eye corner. It is necessary to arrange the patient's surgical position appropriately to ensure a smooth operation. Diabetes insipidus is one of the most common complications associated with pituitary surgery. The nurses should assist patients to indwell a suitable urinary catheter and carefully record the patient's urine output during surgery, which can serve as a reference for doctors' treatment in the future [13].

An important aspect of surgical care is that the hand-washing nurse should be familiar with the steps of the procedure and be able to fully cooperate with the surgeon. During the hemostasis packing gauze after the operation, nurses should pay particular attention to prevent the occurrence of subcutaneous hematoma of the nasal mucosa.

### 3.3. Postoperative

It is important that the nursing staff turn the patient's head to the side before he or she awakens from general anesthesia, to prevent airway obstruction caused by vomiting. As soon as the patient awakens from general anesthesia, help him or her to assume a semirecumbent position and raise his or her head, which can effectively prevent cerebral edema by improving intracranial venous return [14]. Nursing staff should also monitor the patient's body for signs of complications after the operation. Patients should be told that if they find themselves with a large amount of clear liquid in the nasal cavity again, they should seek medical attention at the earliest opportunity and return to the hospital for regular reexaminations to understand how the tumor has changed.

### 3.4. Outcomes

#### 3.4.1. Indicators of Postoperative Recovery

Postoperative hepatic portal exhaust time, bowel sound recovery time, and hospitalization time are among these indicators. Each of these indicators was tracked by the hospital's medical staff [15, 16].

#### 3.4.2. SAS and SDS Scores

Both scales have 20 items each with a total score of 100, with 50–70 being mild anxiety/depression, 71–90 being moderate anxiety/depression, and >90 being severe anxiety/depression. The score is proportional to the degree of anxiety/depression, i.e., the higher the score, the higher the degree of anxiety/depression of the patient.

#### 3.4.3. Contentment

The “Satisfaction Questionnaire” created by the hospital is used to assess the patient's satisfaction. It contains 20 questions. Patients are graded based on their satisfaction with the hospital's various services. Five points are awarded for each question, and the total score is divided as follows: <70 points indicate dissatisfied, 70–89 points indicate satisfied, and ≥90 points indicate very satisfied.

#### 3.4.4. Comfort

The patient's comfort was evaluated using a simplified comfort scale. The scale consists of four dimensions: psychology, physiology, social culture, and environment on a scale of 100 points, ≥90 points are very comfortable; 60–90 points are general comfort; <60 points are discomfort.

#### 3.4.5. Postoperative Complications

Diabetes insipidus, cerebrospinal fluid rhinorrhea, decreased vision, and infection are possible complications of surgery.

### 3.5. Statistical Analysis

SPSS 20.0 software was used as the data analysis software, measurement data were expressed as $\left(\bar{x}\pm s\right)$, and independent *t*-test samples were used to examine the difference; enumeration data were expressed as the number of cases (%), and the test was used to analyze the difference. Statistical significance was set at a *P* value of less than 0.05.

## 4. Results

### 4.1. General Data

In terms of overall baseline data, there was no significant difference between the two patient groups (*P* > 0.05), Table 1.

### 4.2. Comparison of Indices Related to Postoperative Recovery

Patients in the stage group spent considerably less time than those in the routine group to attain postoperative recovery-related indicators (*P* < 0.05), Table 2.

### 4.3. Anxiety (SAS) Depression (SDS) Score Comparison

After therapy, patients in the stage group had substantially lower SAS and SDS levels than those in the routine group (*P* < 0.05), Table 3.

### 4.4. Satisfaction Comparison

After therapy, there was a substantial difference in patient satisfaction between the stage group and the regular group (*P* < 0.05), Table 4.

### 4.5. Comparison of Comfort

Those in the stage group reported considerably higher levels of satisfaction after therapy than patients in the routine group (*P* < 0.05), Table 5.

### 4.6. Comparison of Postoperative Complications

Postoperative complications were much fewer in the stage group (*P* < 0.05), Table 6.

## 5. Discussion

The pituitary tumor is a benign intracranial tumor that is more common in young and middle-aged people; pituitary tumors impact patients' fertility, work, life, and studies to varying degrees. Neuroendoscopic transsphenoidal excision is now one of the most often used treatments for pituitary tumors. This approach has several advantages, including reduced stress on the patient's body, faster recuperation following surgery, and increased patient comfort [17]. Scholars have found that patients with pituitary tumors treated surgically may face a number of postoperative problems, and these issues will have a significant impact on patients' postoperative rehabilitation.

In traditional Chinese medicine, there is no clear record of this disease, but according to clinical observations, the disease is located in the brain, and in traditional Chinese medicine, “brain tumor” can be manifested as such symptoms. At present, the methods of differentiating and treating this disease are inconsistent, and the representative one is Professor Zhang Qiujuan who treats pituitary tumors from phlegm, blood stasis, and the kidney. Chui Ning Fang is a clinical protocol for the treatment of pituitary tumors, and its prescription has also achieved wide recognition from the majority of doctors and patients [18]. In addition, people's expectations for nursing services have risen in recent years as the quality of life has improved [19]. Some experts believe that early implementation of scientific rehabilitation nursing plans after cancer surgery can improve blood circulation and neurotrophic state, reduce postoperative swelling, and improve the state of limb dysfunction [20]. Taking targeted rehabilitation nursing measures is conducive to promoting the recovery of limb function after cancer surgery and to the gradual improvement of the quality of life. It can also promote patients to take staged functional exercise in the early stage, which can promote functional recovery and improve exercise endurance and the quality of life, and the outcome is remarkable [21, 22]. The Chinese medicine nursing program emphasizes the guiding ideology of the holistic view of traditional Chinese medicine and nursing based on syndrome differentiation and always guides the clinical practice with the holistic view of traditional Chinese medicine. The methods of “different nursing for the same disease” and “same nursing for different diseases” are adopted to carry out syndrome-differentiated nursing from the aspects of daily life, diet, emotion, medication, and nursing [23]. Despite the fact that routine nursing interventions such as diet and psychology are included in the routine nursing of neuroendoscopic transsphenoidal pituitary tumor resection, the effect of routine nursing is relatively low due to the insufficient understanding of the time when the patient requires nursing [24].

A staged nursing intervention was used in this trial and has the benefit of allowing matching symptomatic nursing measures for patients' psyche and physiology in various clinical phases. Patients are more prone to suffer fear and anxiety before surgery due to their hazy comprehension of sickness and operation [25], psychological support is therefore necessary at this time. Early on, the nursing staff should pay more attention to the nutritional supplement of the patient's body. After the patient has undergone surgery, if the procedure has been successful, the nursing staff should concentrate on patient observation and preventative measures [26]. This study found that the recovery-related indicators of patients in the staged nursing group were significantly lower than those in the routine group, which indicated that staged nursing could be an effective tool for promoting the postoperative recovery of patients undergoing pituitary tumor resection. Possibly, this is due to the staged nursing preparing the patient's intraoperative posture before surgery, which may result in a reduction of the patient's negative emotions caused by postural discomfort, as well as a reduction of postoperative vomiting; therefore, it is capable of promoting the recovery of patients following surgery.

It has been shown that patients with pituitary tumors are frequently influenced by variables such as sickness, surgery, and strange surroundings in the hospital, which can cause psychological discomfort such as worry and panic, impacting the patient's follow-up therapy [27]. It has been demonstrated by Wang Qin et al. that staged nursing mode intervention can effectively improve the negative emotions of patients and thereby enable them to maintain a positive treatment attitude [28]. According to the results of this study, the SAS and SDS scores of the patients in the stage group after treatment were significantly lower than those of the patients in the routine group, indicating that the staged nursing model intervention could effectively reduce anxiety and depression among patients undergoing pituitary aneurysmectomy. It may be the case that staged nursing mode intervention provides more comprehensive psychological counseling and knowledge explanations to the patients before surgery, facilitating their understanding of their diseases and the operation, thereby alleviating their anxiety [29].

Furthermore, the results of this study revealed that patients in the stage group were significantly more satisfied and comfortable after treatment than those in the routine group, indicating that staged care could significantly improve patient comfort and satisfaction following pituitary tumor resection. The reason for this could be that nurses who practice staged nursing show complete respect and understanding, pay close attention to the physical and psychological changes of patients, and help patients solve the problems they encounter appropriately; as a result, the body and mind reached a state of comfort, which greatly improved the patient's level of satisfaction and comfort [30]. A primary focus of nursing is the management of postoperative complications resulting from pituitary tumors, which not only requires nurses to master the knowledge, skills, and procedures of routine nursing but also requires them to comprehend the pathogenesis and clinical manifestations of postoperative complications [31]. As a result of this complete understanding, the nursing staff will be able to closely observe the occurrence of various complications in the body of the patient following surgery. After neuroendoscopic transsphenoidal pituitary tumor resection, the most commonly reported postoperative complications are diabetes insipidus, rhinorrhea caused by cerebrospinal fluid, impaired vision, infection, etc. It is anticipated that these complications will adversely affect the subsequent rehabilitation of patients [32]. The results of this study demonstrated that the incidence of postoperative complications in patients in the stage group was significantly lower than that in the routine group. This confirms that staged care can effectively reduce the incidence of postoperative complications in patients undergoing pituitary tumor resection. Presumably, this is due to the fact that staged care will employ strict aseptic procedures and will actively take measures such as anti-infection measures and cooling during the surgery, which further reduces the incidence of postoperative complications in patients [33].

The staged nursing path helps reduce the psychological stress of patients. Surgery, as an invasive treatment, is an extremely major source of stress for patients with bad psychological emotions, which can cause different degrees of tension, anxiety, and restlessness in patients undergoing surgery. Patients maintain a good psychological condition before surgery, reduce stress response, and facilitate postoperative recovery. Therefore, the use of staged care, through prehospital assessment to understand the needs of patients, and individualized preoperative health education and psychological care can alleviate the patient's negative psychological emotions and improve the patient's confidence in treatment.

However, there is a limitation in generalizing to disease due to the results of the small number of participants. In addition, the intervention time might not be enough. Thus, further studies are suggested to secure a larger population of subjects with a longer intervention time to counter the limitations.

In summary, staged nursing has a significant effect on patients undergoing neuroendoscopic transsphenoidal pituitary tumor resections. The nursing procedure for this procedure can ensure a smooth completion of the operation, promote the postoperative recovery of patients, and reduce anxiety and depression among patients. In addition, it is guaranteed to reduce the probability of postoperative complications for patients, and its nursing method can also be effectively used to improve the clinical satisfaction and comfort of patients, so its use in clinical practice is highly recommendable.

## Figures and Tables

**Table 1:** Comparison of general data.

	Routine group (*n* = 44)	Stage group (*n* = 44)	*t*/*x*^2^	*P*
Gender			0.192	0.661
Male	26	28		
Female	18	16		

Age (years)	30–52	31–53		
Average age (years)	41.28 ± 5.73	41.37 ± 5.82	−0.073	0.942
Disease duration (months)	2–7	1–7		
Average disease duration (months)	4.23 ± 1.12	4.31 ± 1.20	−0.323	0.747

**Table 2:** Comparison of postoperative recovery-index indicators $\left(\bar{x}\pm s\right)$.

Group (number of cases)	Postoperative hillar exhaust time (h)	Bowel sounds recovery time (h)	Length of hospital stay (d)
Routine group (*n* = 44)	23.66 ± 2.06	16.38 ± 2.42	8.34 ± 2.06
Stage group (*n* = 44)	16.31 ± 1.47	11.21 ± 1.05	5.18 ± 1.05
*t*	19.265	13.0	9.066
*P*	<0.001	<0.001	<0.001

**Table 3:** Anxiety (SAS) depression (SDS) score comparison $\left(\bar{x}\pm s\right)$.

Group	Number of cases	SAS (points)		SDS (min)	
		Before nursing	After nursing	Before nursing	After nursing
Routine group	44	69.35 ± 2.36	58.63 ± 2.57	64.34 ± 3.21	55.62 ± 5.78
Stage group	44	69.41 ± 2.29	48.42 ± 2.67	64.40 ± 3.25	46.51 ± 5.49
*t*	—	−0.121	18.275	−0.087	7.58
*P*	—	0.904	<0.001	0.931	<0.001

**Table 4:** Satisfaction comparison [*n*(%)].

Group	Number of cases	Dissatisfied	Satisfied	Very satisfied	Total satisfaction rate
Routine group	44	15	16	13	29 (66%)
Stage group	44	3	17	24	41 (93%)
*x * ^2^	—	—	—	—	10.057
*P*	—	—	—	—	0.002

**Table 5:** Comparison of comfort [*n*(%)].

Group	Number of cases	Very comfortable	General comfort	Uncomfortable	Total comfort
Routine group	44	11	18	14	30 (68%)
Stage group	44	22	19	3	41 (93%)
*x* ^2^	—	—	—	—	8.822
*P*	—	—	—	—	0.003

**Table 6:** Comparison of postoperative complications [*n*(%)].

Group	Number of cases	Diabetes insipidus	Cerebrospinal fluid rhinorrhea	Vision loss	Infection	Overall incidence (%)
Routine group	44	3	2	2	3	10 (23%)
Stage group	44	1	0	0	1	2 (5%)
*x* ^2^	—	—	—	—	—	6.175
*P*	—	—	—	—	—	0.013

## Data Availability

No data were used to support this study.
